RETRACTED

# PASS-Predicted Hepatoprotective Activity of *Caesalpinia sappan* in Thioacetamide-Induced Liver Fibrosis in Rats

**DOI:** 10.1155/2014/301879

**Published:** 2014-02-20

**Authors:** Farkaad A. Kadir, Normadiah M. Kassim, Mahmood Ameen Abdulla, Behnam Kamalidehghan, Fatemeh Ahmadipour, Wageeh A. Yehye

**Affiliations:** ^1^Department of Anatomy, Faculty of Medicine, University of Malaya, 50603 Kuala Lumpur, Malaysia; ^2^Department of Biomedical Science, Faculty of Medicine, University of Malaya, 50603 Kuala Lumpur, Malaysia; ^3^Department of Pharmacy, Faculty of Medicine, University of Malaya, 50603 Kuala Lumpur, Malaysia; ^4^Nanotechnology & Catalysis Research Centre (NANOCAT), University of Malaya, Block 3A, Institute of Postgraduate Studies Building, 50603 Kuala Lumpur, Malaysia

## Abstract

The antifibrotic effects of traditional medicinal herb *Caesalpinia sappan* (CS) extract on liver fibrosis induced by thioacetamide (TAA) and the expression of transforming growth factor **β**1 (TGF-**β**1), **α**-smooth muscle actin (**α**SMA), and proliferating cell nuclear antigen (PCNA) in rats were studied. A computer-aided prediction of antioxidant and hepatoprotective activities was primarily performed with the Prediction Activity Spectra of the Substance (PASS) Program. Liver fibrosis was induced in male Sprague Dawley rats by TAA administration (0.03% w/v) in drinking water for a period of 12 weeks. Rats were divided into seven groups: control, TAA, Silymarin (SY), and CS 300 mg/kg body weight and 100 mg/kg groups. The effect of CS on liver fibrogenesis was determined by Masson's trichrome staining, immunohistochemical analysis, and western blotting. *In vivo* determination of hepatic antioxidant activities, cytochrome P450 2E1 (CYP2E1), and matrix metalloproteinases (MPPS) was employed. CS treatment had significantly increased hepatic antioxidant enzymes activity in the TAA-treated rats. Liver fibrosis was greatly alleviated in rats when treated with CS extract. CS treatment was noted to normalize the expression of TGF-**β**1, **α**SMA, PCNA, MMPs, and TIMP1 proteins. PASS-predicted plant activity could efficiently guide in selecting a promising pharmaceutical lead with high accuracy and required antioxidant and hepatoprotective properties.

## 1. Introduction

Liver fibrosis is known to result in distortion of normal tissue architecture of the liver. This alteration resulted from chronic liver damage as seen in chronic alcoholic abuse, viral hepatitis, or inherited metabolic disease [1]. Several biological and biochemical disturbances may also lead to hepatic cirrhosis [2]. A fibrotic liver may contain a substantial increase in most of the matrix proteins, in particular, the interstitial collagen types I and III which are under the influences of cytokines like transforming growth factor beta 1 (TGF-*β*1) and *α*-smooth muscle actin (*α*SMA) [3, 4]. These cytokines not only are present in greater amounts but also are deposited in abnormal sites within the liver microanatomy [5]. In case of thioacetamide- (TAA-) induced liver cirrhosis, other parameters such as oxidative stress have been postulated to be major molecular mechanisms basic to tissue alteration [6].

RETRACTED

*Caesalpinia sappan *(CS), commonly named as Brazil or Sappan, belongs to the family of Caesalpiniaceae, a native plant in Southeast Asia [7]. Several studies have shown that CS has antimicrobial and bactericidal activity [8] and antiallergic [9], neuroprotective [10], and hypoglycaemic effects [11]. Others found that extract from CS can be used for treating ascites, tumour, leukaemia [12], and arteriosclerosis [13]. This could be due to its antioxidant activity and its capability to inhibit malondialdehyde (MDA) and scavenging of superoxide anions, hydrogen peroxide, and hydroxyl radicals [14]. In another instance, the methanolic and aqueous extracts of CS showed hepatoprotective effect against CCl_4_ and acetaminophen induced liver damage in experimental animals [15, 16]. Thorough screening is necessary to understand the pharmacological action of the plant compounds [17].

The prediction of activity spectra for substances (PASS) software [18], which predicted more than 300 pharmacological effects and biological and biochemical mechanisms based on the structural formula of the substance, was efficiently used in this study to reveal new multitalented actions of the isolated components of CS extract. In order to investigate further whether CS has a preventive effect on liver fibrogenesis and how it works, this study was designed to examine the pathological changes of liver fibrosis with and without CS treatment.

TGF-*β*1, a crucial cytokine, plays an essential role in the progression of liver cirrhosis by its dominant activation on the hepatic stellate cells (HSC_S_). This action is accompanied by a loss of cellular retinoid, increase synthesis of *α*-smooth muscle actin (*α*SMA) and large quantities of the major components of the ECM, including collagen types I, III, and IV, fibronectin, and laminin [4, 19]. We strongly believe that antioxidants are able to reduce hepatic inflammation and fibrosis, thus slowing or even preventing the progression to cirrhosis. Therefore, based on this action, we hope to show that CS is beneficial for the treatment of liver fibrosis, possibly arbitrated through the downregulation of TGF-*β*1 and *α*SMA.

RETRACTED

## 2. Materials and Methods

### 2.1. Computational Evaluation of Biological Activity

The biological activity spectra of the isolated compounds for CS extract were obtained using the Prediction of Activity Spectra for Substances (PASS) software. PASS prediction tool is constructed using 20,000 principal compounds from the MDDR database (produced by Accelrys and Prous Science) [20].

### 2.2. Preparation of Crude Ethanol Extract

Fresh leaves of CS plant were obtained from Kampung Baru, Sungai Ara, Penang, Malaysia. The plant was identified, and the voucher specimen number (KLU 47313) was kept in University of Malaya (Department of Pharmacy). The plant was dried and ground to fine powder, after that homogenized in 95% ethanol at a ratio of 1 : 10 of plant to ethanol, and left to soak for four days at 25°C with occasional shaking and stirring. Next, the mixture was filtered using a filter paper, and the resulting liquid was concentrated at reduced pressure at 45°C to obtain a dark gummy-green extract. The extract was then dissolved in Tween 20 (10% w/v) and administered orally to rats in concentrations of 100 and 300 mg/kg body weight.

### 2.3. Preparation of TAA

TAA (Sigma-Aldrich, Switzerland) and all other chemicals used were of analytical grade and purchased mostly from Sigma-Aldrich and Fisher. TAA stock solution of 5 gm/L was prepared by dissolving the pure TAA which is in the crystal form in distilled water, 0.03% w/v TAA solution. This mixture was given to the rats as their daily drinking water.

### 2.4. Preparation of Silymarin (SY)

SY (International Laboratory, USA), a well-known standard drug with hepatoprotective activity, was used as a standard drug in this study. It was dissolved in Tween 20 (10% w/v) and orally administered to rats in concentrations of 50 mg/kg body weight [6].

### 2.5. Animals

Adult male healthy *Sprague Dawley *(SD) rats weighing 180–200 gm were obtained from Animal House Unit, Faculty of Medicine, University of Malaya, Malaysia. They were kept in wire-bottomed cages at 25 ± 3°C temperature, 50–60% humidity, and a 12 h light-dark cycle for at least a week before the experiment. They were maintained under standard housing conditions and free access to standard diet and water ad libitum during the experiment. The experimental protocol was approved by Animal Ethics Committee, with an ethical number ANA/18/05/2012/FAAK. Throughout the experiments, all criteria of taking care of animals prepared by the National Academy of Sciences and outlined in the “Guide for the Care and Use of Laboratory Animals” were applied [21].

The animals were randomly divided into seven groups of six rats each and treated as follows. Group 1: normal control—rats were administered orally with 10% Tween 20 (5 mL/kg) daily. Group 2: TAA group—rats were given 0.03% TAA with their drinking water daily. Group 3: SY group—rats were given SY 50 mg/kg orally + 0.03% TAA daily. Group 4: low dose CS group—rats were given CS100 mg/kg orally. Group 5: low dose CS + TAA group—rats were given CS100 mg/kg orally + 0.03% TAA daily, Group 6: high dose CS group—rats were given CS300 mg/kg orally. Group 7: high dose CS + TAA group—rats were given CS300 mg/kg orally + 0.03% TAA daily. The experiment was carried out for a total duration of 12 weeks.

RETRACTED

At the end of the twelve-week period, the rats were anaesthetized by intramuscular injection of 50 mg/kg ketamine mixed with xylazine 5 mg/kg. 24 hours after the last treatment and overnight fasting, laparotomy was done, livers and spleens were washed quickly *in situ* with ice-cold isotonic saline and harvested, and parts of the liver were carefully divided into four portions: two portions from the right lobe, one for histological and the other for immunohistochemical examination. Each was fixed with formalin and processed for light microscopy within three days. The 3rd and 4th portions were taken from the left lobe and stored at −80°C until used for western blot analysis and detection of endogenous antioxidant enzymes, hepatic CYP2E1 level, and matrix metalloproteinase enzymes (MMP-2, MMP-9, and TIMP-1).

#### 2.5.1. Histopathological Study

The right lobes of liver samples from rats of all groups were fixed in 10% buffered formalin solution, processed by light microscopy by paraffin slice technique. Sections with 5 *μ*m thickness were stained with special stains (Masson's trichrome) for collagen. Each section was subjectively scored by two blinded experienced observers, including an anatomist and a histopathologist for evidence of fibrosis, fatty change, architectural distortion, and regenerative nodules. The extent of bile duct proliferation and fibrosis was duly graded by a semiquantitative method on a scale between zero and six [22]. Stage 0 values were indicative of normal liver architecture in which there was no evidence of bile duct proliferation, inflammation, and fibrosis, whereas stage 6 reflected a gross destruction of the hepatic architecture typified by marked proliferation of the bile ducts with severe inflammation and a very conspicuous fibrotic response (Table 2). Each sample was observed under 10x magnification power. The degree of fibrosis was expressed as the mean of 10 different fields in each slide [23]. The histology of the livers from CS-treated rats was compared to that of the TAA control group. This comparison was to determine the effect of the herbs in TAA-treated groups.

RETRACTED

#### 2.5.2. Immunohistochemical Localization of TGF-*β*1 in Rat Liver and PCNA in Rat Spleen

Mouse monoclonal [2Ar2] to TGF *β*1 (100 ug) immunohistochemistry kit (ab64715) (Abcam) and mouse monoclonal Anti-PCNA antibody [PC10] proliferation marker ab29 (Abcam) were used for TGF *β*1 and PCNA determination, respectively. Briefly, by using poly-L-lysine-coated slides, liver and spleen sections were prepared and heated in an oven (Venticell, MMM, Einrichtungen, Germany) for 25 minutes at 60°C. After heating, the sections were deparaffinized in xylene and hydrated in a series of graded alcohol. Antigen recovery procedure was conducted in 10 mM sodium citrate buffer boiled in a microwave. Staining method was conducted following the company's guidelines (DakoCytomation, USA). Briefly, 0.03% hydrogen peroxide sodium azide was used to block the endogenous peroxidase for 5 min. Then sections were carefully washed with clean wash buffer. After washing, the liver sections were incubated with monoclonal antibody of TGF-*β*1 (diluted to 1 : 50) at 37°C for 60 min and spleen sections were incubated with (PCNA) (1 : 200) biotinylated primary antibodies for 15 minutes. Following gentle washing with wash buffer, the sections were reincubated for 15 min with streptavidin HRP. Then, the sections were incubated with diaminobenzidine substrate chromogen for over 7 min followed by washing and counterstaining with hematoxylin for 5 seconds. Tissue sections were finally dipped 5 times in ammonia (0.037 mol/L), cleaned, and covered with cover slip. Sections were viewed under a microscope to examine the presence of cytoplasmic brown granules for the positive expression of TGF-*β*1 and brown-stained nuclei for positive expression of PCN antigens.

Two blinded experienced observers, including an anatomist and a histopathologist confirmed the immunohistochemical analysis. The histology of the livers from each group of herb-treated rats was compared to the normal and TAA groups. These comparisons were to confirm the effect of the herb in TAA-treated groups.

#### 2.5.3. Western Blot Analysis of TGF *β*1 and *α*SMA Expression

An analytic technique was used to detect specific proteins in a given sample of tissue, homogenate, or extract. Identification is based upon the transfer of proteins from a gel (polyacrylamide gel) to polyvinylidene difluoride membrane (PVDF) or nitrocellulose membrane and eventually detecting a target protein based on its property to specifically bind to an antibody.

The protein is usually separated by SDS page based on the size of protein particles using electrophoresis and then followed by blotting the protein onto a membrane by probing with antibodies. It is important to transfer the proteins to the membranes from gels for the efficient binding to the probe antibody as polyacrylamide gel is not particularly amenable to the diffusion of large molecules. The attachment of specific antibodies to specific immobilised antigens onto the membrane can be readily visualized by indirect enzyme immunoassay techniques, usually using a chromogenic substrate which creates an insoluble product. This analysis was used to investigate the expression of fibrosis-related proteins, including TGF-*β*1 (ab64715), Abcam, and *α*SMA (ab5694) (Abcam).

RETRACTED

Briefly, livers were homogenized in ice-cold lysis buffer (50 mM Tris-HCL (pH 8.0), 120 mM NaCl, 0.5% NP-40, 1 mM PMSF). Lysates were centrifuged at 14,800 g for 30 min, and aliquots of supernatant containing 30 *μ*g proteins were boiled in a sodium dodecyl sulphate (SDS) sample buffer for 5 min before electrophoresis in 10% SDS-polyacrylamide gel. After electrophoresis, proteins were transferred to a polyvinylidene difluoride membrane (PVDF) (Bio-Rad, USA) using the semidry transfer unit (Hoefer TE 70X, USA), and the blots were blocked with 5% nonfat milk in TBS-Tween buffer (0.12 M Tris-base, 1.5 M NaCl, and 0.1% Tween 20) for 1 hour at room temperature and then washed in PBST buffer. The primary antibodies TGF-*β*1 (1 : 2000), *α*SMA (1 : 13 5000) were purchased from Abcam and *β*-actin (1 : 2000) Santa Cruz Biotechnology, Inc., CA, USA, which was used as an internal control were incubated with the membranes at 4°C overnight. Followed by the incubation for 1 hour at room temperature with goat anti-mouse and goat anti-rabbit secondary antibodies conjugated with alkaline phosphatase (i-DNA, USA) at a ratio of 1 : 1000 and then washed twice with TBST for 10 minutes three times on an orbital shaker. Then, blots were developed using the BCIP/NBT (Santa Cruz, USA) solution for a period of 5–30 minutes to detect the target protein band as a precipitated dark-blue colour.

#### 2.5.4. Antioxidant Activity

Liver samples were washed immediately with ice-cold saline to remove excess blood. Liver homogenates (10% w/v) were prepared in cold 50 mM potassium phosphate buffer saline (PBS) (pH 7.4) using homogenizer in ice. The cell debris was removed by centrifugation at 4500 rpm for 15 min at 4°C using a refrigerated centrifuge Rotofix 32 (Hettich Zentrifugen, Germany). The supernatant was used in the estimation of the following *in vivo* antioxidant using commercially available kits (Cayman Chemical Company, USA): catalase (CAT) (item number 707002), superoxide dismutase (SOD) (item number 706002), and glutathione peroxidase (GPx) (item number 703102) activities. All assays were performed according to the instruction manual of the manufacturer.

RETRACTED

#### 2.5.5. Assessment of Hepatic Cytochrome P450 2E1 (CYP2E1) Level

To demonstrate the effect of the CS extract on the level of CYP2E1 as an important enzyme in the biotransformation of TAA in the liver microsome [24], the tissue homogenate from all rats was tested for the level of CYP2E1 enzyme by following the instructions of Uscn Life Inc. (SEA988Ra, China). Briefly, 100 *μ*L of the sample was incubated with precoated capture antibody specific to CYP2E1 in duplicate in 96-well plate for 2 hours at 37°C. After brief rinsing, the sample was incubated for 1 hour at 37°C with 100 *μ*L of biotin-conjugated secondary antibody followed by three-time washing using 350 *μ*L washing buffer (1x). 100 *μ*L streptavidin-horseradish peroxidase (HRP) was added to the sample and incubated for 30 minutes at 37°C followed by 5 repeated washes. 90 *μ*L tetramethylbenzidine (TMB) was added in the sample as a colorimetric reagent and incubated for 20 minutes. Finally, the reaction was stopped using 50 *μ*L of H_2_SO_4_ and the absorbance was read at 450 nm.

#### 2.5.6. Evaluation of Matrix Metalloproteinase Enzymes (MMP-2 and MMP-9) and TIMP-1

Matrix metalloproteinase enzymes (MMP-2 and MMP-9) and their partial regulator tissue inhibitor of metalloproteinase (TIMP-1) play a role in liver damage [25]. For this purpose, the following assay was conducted to demonstrate the effect of CS extract on these enzymes in the liver tissue homogenate collected from the rats of all groups as mentioned previously and assayed in duplicate by enzyme-linked immunosorbent assay kit following the manuals by the manufacturer (Uscn Life Science SEA551Ra, SEA553Ra, and SEA552Ra, China), respectively.

### 2.6. Statistical Analysis

The results were presented as mean ± standard error of mean. The one-way ANOVA test with post hoc test using Bonferroni multiple comparisons in the PASW program (version 18) for Windows (SPSS Inc., Chicago, IL, USA) was used to analyse the data, with *P* < 0.05 being considered as the limit of significance.

## 3. Results

### 3.1. PASS Prediction and Assistant Experimental Design

A computed study using PASS program of CS extract isolated compounds of lipid peroxidase inhibitor, antioxidant, free radical scavenger, and hepatoprotectant is given in Table 1. The highest hepatoprotective activity belonged to sappanchalcone with pa 92% compared to the other constituents. Similarly, sappanchalcone also revealed the highest antioxidant, radical scavenging, and lipid peroxidation inhibition activities giving pa 83%, 95%, and 81%, respectively.

### 3.2. Histopathological Findings of the Liver

Livers from the normal, CS100, and CS300 groups showed normal lobular architecture with distinct hepatic cells, sinusoidal spaces, and a central vein. On the other hand, the livers of the TAA-treated animals exhibited loss of normal lobular architecture with the presence of regenerating nodules separated by fibrous septa extending from the central vein. There were some inflammatory cells, abnormal appearance of portal tracts, and twinning of the cell plates. This morphological appearance could be due to regenerating activity of the hepatocytes which contained cytoplasmic vacuolation. There were fatty changes, sinusoidal dilatation, proliferation of bile duct, and centrilobular necrosis as well as bundles of collagen surrounding the lobules, which resulted in huge fibrous septa and distorted tissue architecture. The cirrhotic nodules which were shown by using Masson's trichrome staining revealed thick green bundles of collagen which appeared and separated the regenerative nodules (Figure 1).

RETRACTED

Histopathological examination of livers of CS-treated animals showed good recovery of TAA-induced fibrosis as compared to SY. Animals treated with the higher dose of the extract showed remarkable histological regeneration compared to those of the low dose group. They showed nearly ordinary patterns with an increase normal hepatocytes parenchyma and a reduced development of fibrous septa and lymphocytes infiltration (Figure 1).

### 3.3. Immunohistochemistry of TGF-*β*1

TGF-*β*1 staining of hepatocytes from the livers of CS-treated groups is shown in (Figure 2). Hepatocytes of liver tissues from TAA-group rats showed upregulation of TGF-*β*1 staining accompanied with downregulation in the normal control group. Hepatocytes from SY-treated rats showed downregulated TGF-*β*1 expression, which suggested lower levels of fibrosis. Liver tissues treated with high dose CS extract inhibit hepatocyte fibrosis as indicated by downregulated TGF-*β*1 expression, while the low dose CS extract still showed moderate expression for TGF-*β*1 within the hepatocytes and near the central vein areas. These findings support the idea of CS extract-induced hepatoprotective activities against progressive liver damage by inhibiting fibrosis of hepatocytes and ameliorating their proliferation.

Splenic tissues from TAA-treated rats revealed high expression of PCNA staining indicating severe necrosis as evidenced by high cellular proliferation in the attempt to repair the damaged spleen. In contrast, the spleens from SY as well as the low dose and high dose CS-treated rats showed less expression of PCNA staining indicating lower degree of necrotised hepatocytes proliferation than of apoptosis (Figure 3).

RETRACTED

### 3.4. Expression of TGF-*β*1 and *α*SMA by Western Blot Analysis

Remarkable TGF-*β*1 and *α*SMA expression was observed in TAA group and decreased in SY + TAA group. In groups 4 and 5 western blot analysis revealed slight TGF-*β*1 and *α*SMA expression (Figure 4).

The treatment of liver fibrosis with CS300 + TAA reduced the expression of TGF-*β*1 and *α*SMA in a level comparable with SY + TAA. However, the low dose CS100 + TAA was not as effective as SY + TAA (Figure 5).

### 3.5. *In Vivo* Antioxidant in Liver Tissue Result

CAT, SOD, and GPx are some of the components of the intrinsic antioxidant defence system enzymes which were significantly (*P* < 0.05) increased in high dose treatment groups CS and SY but decreased in TAA-induced groups due to long term excretion of free radicals as shown in (Table 3).

### 3.6. Hepatic CYP2E1 Levels

The result of the effect of CS extract on the hepatic cytochrome enzyme CYP2E1 is shown in Figure 6. Animals from the cirrhosis control group had significantly (*P* < 0.05) higher levels (3.32 ± 0.87 ng/mL) of CYP2E1 compared with normal group (1.64 ± 0.62 ng/mL) and SY-treated group (1.76 ± 0.51 ng/mL). On the other hand, there was no significant difference between the low dose and high dose of the CS-treated animals which had similar CYP2E1 levels (2.72 ± 0.37 and 2.53 ± 0.52 ng/mL resp.) in comparison with the normal control and cirrhosis groups.

### 3.7. Hepatic MMP-2, MMP-9, and TIMP-1

The effects of CS extract treatment on the liver tissue level of MMP-2, MMP-9, and TIMP-1 collected from all experimental animals are illustrated in Table 4. It was noted that the levels of the tested enzymes were significantly high (*P* < 0.05) in the cirrhosis control group rats compared to all other groups. On the other hand, administration of CS extract to the animals significantly (*P* < 0.05) attenuated the enzymatic level of MMP-2, MMP-9, and TIMP-1 to approach the values of the reference or standard control group (SY + TAA), which indicates the efficacy of the plant extract treatment in a dose-dependent manner. Furthermore, oral administration of low and high doses of CS reduced the hepatic MMP-9 level to approach the values of SY-treated group.

## 4. Discussion

Oxidative stress and its consequent lipid peroxidation have been currently considered to be involved in the generation of TAA-induced cirrhosis [26]. Soon after its administration, TAA is converted to TAA-S oxide (TASO) by the mixed function oxidase system. TASO is subsequently transformed into thioacetamide S, S-dioxide with or without being further oxidized to form species that exert their toxic effect on several organs, including plasma, liver, kidney, bone marrow, adrenals, and other tissues. TAA undergoes an extensive metabolism to acetate, and it is finally excreted through the urine within 24 hours [27]. These changes lead to cell injury, and chronic liver injury leads to excessive deposition of collagen in the liver, resulting in liver fibrosis [28].

RETRACTED

Liver cirrhosis is a major disease associated with various pathological processes, including progressive fibrosis, portal hypertension, and carcinoma [29]. Many liver protective and antifibrotic agents from natural products have been used in traditional medicine for the treatment of liver diseases [30–34]. In order to accelerate the search for potent natural products, computer-aided drug discovery program PASS was used to predict the antioxidant and hepatoprotective properties of CS isolated compounds. PASS prediction tools are constructed using 20000 principal compounds [35] and about 4000 kinds of biological activity based on the structural formula with mean accuracy about 90% [36]. The result of prediction is presented as the list of activities with appropriate Pa and Pi ratio (Table 1). Pa and Pi are the estimates of probability for the compound to be active and inactive, respectively.

It is reasonable that only those types of activities may be revealed by the compound, in which Pa > Pi. If Pa > 0.3 the compound is likely to reveal this activity in experiments, but, in this case, the chance of being the analogue of the known pharmaceutical agents for this compound is also high. Thus, the potential biological effects of the plant constituents were predicted by PASS program based on structure activity relationship (SAR) analysis of the training set containing thousands of compounds, which have many kinds of biological activity. Therefore, before we started our experiments, we used PASS program to validate whether CS constituents based on SAR strategy is in agreement with the SAR of the training set of the PASS database.

CS leaves are inexpensive and widely available and they showed potential in treating diabetes mellitus [37], arteriosclerosis [38], ascites, tumour, and leukaemia [12] in part owing to its potent antioxidant properties [14]. Basic research has found that CS extract has a protective effect on hepatic endothelial cells and microcirculation in rats with chronic liver injury induced by CCl_4_ [15] and acetaminophen [16]. This property could be due to the presence of several phenolic compounds, flavonoids, and brazilin, a major constituent as hepatoprotective agent.

Our results showed that the levels of TGF-*β*1 and *α*SMA did not change in the normal control group (Figures 2 and 4). This finding supports the idea that the hepatic satellite cells (HSCs) were still in their quiescent state. However, these HSCs were activated in the presence of TAA leading to high production of ECM and consequentl, high expression of TGF-*β*1 and *α*SMA. HSCs, being the main cellular source of ECM during chronic liver injury, undergo a transition into *α*SMA expressing myofibroblast-like cells. Activation of HSC is associated with cell proliferation, increased contractility, and enhancement of matrix production [39]. TGF-*β*1 is mainly found in portal tract and fibrous septa where proliferation of the ducts corresponds to the distribution of collagen [40]. This suggests that reactive-oxygen-species-(ROS) induced HSC activation can be inhibited by antioxidants. Based on these findings, our results demonstrate that CS treatment during the development of liver fibrosis managed to reduce *α*SMA expression compared to the hepatotoxic TAA group which showed marked increased *α*SMA expression (Figure 4). This indicates that CS extract has the potential action to suppress HSC activation through inhibition of ROS.

RETRACTED

The three isoforms for TGF-*β* are *β*1,  *β*2, and *β*3. TGF-*β*1 is an important profibrogenic cytokine in liver injury and it is biologically active with multiple pharmacological actions [41]. A balance among these actions is required to maintain tissue homeostasis. The aberrant expression of TGF-*β*1 is involved in the pathogenesis of liver diseases [42]. It is known that TGF-*β*1 is a crucial cytokine which is involved in the early stages of liver fibrosis. Oxidative stress triggers TGF-*β*1, resulting in the latter stimulating ECM production and deposition [42]. Therefore, one of the effective strategies to produce antifibrotic drug is to identify the anti-TGF-*β*1 agents.

Immunohistochemical analysis of TAA liver tissue showed that the cells were positive for TGF-*β*1 in the portal areas and around the central veins. Administration of CS ethanolic extract in TAA-treated rats was noted to downregulate TGF-*β*1 expression (Figure 2), suggesting that CS extract is an effective TGF-*β*1 inhibitor. Our finding supports a previous study [43]. Cellular proliferation is thought to play an influential role in several steps of the carcinogenic process [44]. The detection of PCNA using immunohistochemical methods is a common way to study the proliferating activity of cells. The PCNA indicating the number of regenerating splenic cells parallels the severity of liver cirrhosis (Figure 3). Localized expression of PCNA in areas of high proliferative activity might be an early event in the pathogenesis of hepatic neoplasia which is one of the most common complications of liver cirrhosis.

RETRACTED

In our western blot assay, we observed that TAA increased *α*SMA and TGF-*β*1 expression in the liver which suggests that *α*SMA and TGF-*β*1 could participate in liver injury or as an early reaction of liver cirrhosis (Figures 4 and 5). Interestingly, TAA treatment causes sharp bands to be formed, in contrast to smeared bands in the normal group. Since the internal control (*β* actin) is clearly detected, this result is not due to experimental errors, such as revers transcription failures or RNA degradation [45]. Treating the animals with the CS extract inhibited the necrotic effect due to TAA administration by modifying necrosis into apoptosis, which may be via the cytochrome release from mitochondria and caspase activation [46]. This modification *in vivo* would scale down the release of inflammatory mediators that would prevent progressive liver damage.

There is a possibility that CS might have altered the metabolism of TAA, thereby leading to a less toxic effect. Taking the antioxidant ability of CS [14] and the metabolic characteristics of TAA into account [27], we found that treatment with CS significantly reduced the impact of TAA toxicity, through removing the causative stimuli of TAA, neutralizing the ROS by their high antioxidant content, and attenuating endogenous antioxidant enzymes (CAT, SOD, and GPX) to their normal levels (Table 3). In fact, during oxidative stress, the body uses its defence mechanism to minimize the process of lipid peroxidation by using these antioxidant enzymes. Thus, the activity of those enzymes becomes higher in early stages of TAA induction, but when the insult continues for a long period, the enzymes become depleted and are unable to fight against the free radicals. This means that in advanced stages of peroxidation due to TAA, the activity of CAT, SOD, and GPX was declined, while the levels of these enzymes continue to be high in the treatment groups due to the antioxidant properties of plant extracts against TAA-induced free radicals.

TAA is metabolized by CYP2E1 enzymes in liver microsomes and is converted to toxic reactive intermediate called thioacetamide sulphur dioxide through oxidation [26]. Cytokines and growth factors expressed during liver regeneration are associated with expression of their receptors. Therefore, we measure the level of CYP2E1 inhibition, attenuating drug-induced hepatotoxicity. The inhibiting effect of CS extract to CYP2E1 (Figure 6) may be one of the significant factors in hepatoprotective activity by inhibiting the metabolism of TAA and blocking the release of ROS that is responsible for inducing damage of hepatocytes. Parallel findings were consistent with our study, which showed that *Curcuma longa *possessed protective effect against TAA [47]. ECM is mainly controlled by matrix metalloproteinases (MMPs), which are a group of proteolytic enzymes that are able to degrade the ECM [48, 49]. Tissue inhibitors of metalloproteinases (TIMPs) regulate tightly the activity of MMPs [50, 51]. MMP-9 and TIMP-1 were identified as the molecular signatures during the progress of liver cirrhosis induced by TAA [52]. Park et al., 2010 [45], observed that TAA increased MMP-2 expression in the liver tissues of rats and reported that the balance of MMPs and TIMPs is the key factor of liver fibrogenesis.

RETRACTED

In our research, we studied the effect of CS extract on the level of MMP-2, MMP-9, and TIMP-1 in the rat livers intoxicated with TAA. Our results revealed that administration of CS extract significantly downregulated the levels of MMP-2 and MMP-9 in the rats' livers similar to that of SY, the reference drug used in the study (Table 4). Our results are in agreement with a previous study confirming the hepatoprotective effect of curcumin, the active antioxidant compound of *C. longa *rhizomes [53]. Hence, the extract of CS which suppressed TGF-*β*1 *α*SMA and PCNA expression and reduced the fibrogenesis process could be a promising antifibrotic agent in TAA-induced liver fibrosis. Furthermore, the absence of side effects and a reasonable price may be strong advantages of CS as a choice for alleviating liver fibrosis*.*

## 5. Conclusions

This study demonstrates that CS extract can effectively alleviate liver fibrosis induced by TAA ingestion in rats monitored by marked downregulation of hepatic TGF-*β*1, *α*SMA, and splenic PCNA expression presumably due to the presence of the active component sappanchalcone. Therefore, we suggest that CS can be used as a medicament or food additive for prevention of human liver fibrosis, and future studies could evaluate specifically the hepatoprotective activity of sappanchalcone.

## Figures and Tables

**Figure 1:** Photomicrographs of livers from the different experimental groups: (a) control group: showing normal liver architecture, (b) TAA group (hepatotoxic group): showing proliferation of bile duct and thick fibrous septa, (c) SY + TAA group: showing mild fibrous septa, (d) CS100 group: showing normal liver architecture, (e) CS100 + TAA group: showing multiple nodules with moderate fibrous septa and fewer cirrhotic nodules, (f) CS300 group: showing normal liver architecture, and (g) CS300 + TAA: showing mild fibrous septa. Masson's trichrome stain (Bar scale: 100 *μ*m).

**Figure 2:** Photomicrographs showing immunohistochemistry staining of TGF-*β*1 of livers from the different experimental groups. Control group: showing normal liver architecture, (b) TAA group (hepatotoxic group): showing more TGF-*β*1 expression, (c) SY + TAA group: showing mild TGF-*β*1-positive hepatocytes in the liver, (d) CS100 + TAA group: showing moderate TGF-*β*1 expression, and (e) CS300 + TAA group: showing mild TGF-*β*1 expression. (Bar scale: 50 *μ*m).

RETRACTED

**Figure 3:** Photomicrographs showing immunohistochemical staining of PCNA of spleens from the different experimental groups. Control group: showing normal spleen architecture, (b) TAA group (hepatotoxic group): showing more PCNA expression (white arrows), (c) SY + TAA group: showing mild PCNA positive in the spleen, (d) CS100 + TAA group: showing moderate PCNA expression, and (e) CS300 + TAA group: showing mild PCNA expression. (Bar scale: 10 *μ*m).

**Figure 4:** Western blot analysis of TGF-*β*1 and *α*SMA levels in liver tissue for all experimental groups. (1) Normal control group, (2) TAA group (hepatotoxic group), (3) SY + TAA group, (4) CS100 + TAA group, and (5) CS300 + TAA group.

**Figure 5:** Protein expressions from western blots in all experimental groups are quantitated using Image J program. (a) TGF-*β*1 density. (b) *α*SMA density. The data were stated as mean ± S.E.M. (*n* = 3). Means with different superscripts are significantly different. ^a^ *P* < 0.05 versus normal control group and ^b^ *P* < 0.05 versus TAA control group. SY stands for Silymarin (standard hepatoprotective drug).

**Figure 6:** Effect of CS crude extract on hepatic levels of CYP2E1 in rats at the end of 12 weeks. The data were stated as mean *±* S.E.M. Means with different superscripts are significantly different. ^a^ *P* < 0.05 versus normal control group and ^b^ *P* < 0.05 versus TAA control group. SY stands for Silymarin (standard hepatoprotective drug).

**Table 1:** Part of the predicted biological activities spectra for the chemical compounds of CS extract.

Chemical compounds	Biological activity							
	Lipid peroxidation inhibitor		Antioxidant		Free radical scavengers		Hepatoprotectant	
	Pa	Pi	Pa	Pi	Pa	Pi	Pa	Pi
Protosappanin A	0.495	0.017	0.324	0.019	0.360	0.021	0.264	0.076
Protosappanin B	0.419	0.030	0.416	0.011	0.366	0.021	0.454	0.024
Lyoniresinol	0.355	0.048	0.246	0.037	0.233	0.054	0.383	0.035
(8S,8′S)-Bisdihydrosiringenin	0.415	0.031	0.610	0.004	0.424	0.015	0.434	0.027
Sappanchalcone	0.810	0.003	0.83	0.003	0.95	0.001	0.92	0.002
3-Deoxysappanchalcone	0.655	0.006	0.49	0.007	0.626	0.005	0.590	0.013
Brazilein	0.372	0.043	0.304	0.022	0.440	0.014	—	—
3-Omethybrazilin	0.423	0.029	0.292	0.024	0.733	0.004	0.314	0.055
Brazilin	0.393	0.037	0.293	0.024	0.667	0.004	0.280	0.067
Sappanone B	0.410	0.032	0.377	0.014	0.392	0.018	0.302	0.059
3-Deoxysappanone B	0.445	0.024	0.384	0.014	0.351	0.022	0.288	0.064
3-Deoxy-4-O-methylepisappanol	0.350	0.050	0.276	0.028	0.262	0.041	0.260	0.079

Pa: probability “to be active”; Pi: probability “to be inactive.”

RETRACTED

**Table 2:** Scoring of fibrosis for the different groups.

Group	Pathological staging								Average of stages
	N	0	I	II	III	IV	V	VI	
Normal	6	6	0	0	0	0	0	0	0.0^b^
TAA	6	0	0	0	0	2	2	2	5.00 ± 0.89^a^
SY + TAA	6	0	5	1	0	0	0	0	1.16 ± 0.408^b,a^
CS100 + TAA	6	6	0	0	0	4	2	0	3.33 ± 0.516^b,a^
CS300 + TAA	6	2	4	0	0	0	0	0	0.66 ± 0.51^b^

The data were stated as mean ± S.E.M. Means with different superscripts are significantly different. ^a^ *P* < 0.05 versus normal control group and ^b^ *P* < 0.05 versus TAA control group. SY stands for Silymarin (standard hepatoprotective drug).

**Table 3:** Effect of TAA, SY, and CS ethanolic extracts intake on some *in vivo* antioxidant parameters in TAA-induced liver cirrhosis in rats.

Group	CAT (nmol/min/mL)	SOD (U/mL)	GPx (nmol/min/mL)
Normal	2757.97 ± 49.6^b^	350.84 ± 44.3^b^	141.12 ± 6.89^b^
TAA	2111.42 ± 14.38^a^	218.46 ± 7.48^a^	81.38 ± 4.30
CS100	2666.20 ± 99.9^b^	332.8 ± 23.6^b^	134.2 ± 4.14^b^
CS300	2730.76 ± 40.82^b^	326.8 ± 32.8^b^	136.0 ± 5.78^b^
CS100 + TAA	2424.68 ± 39.04^b,a^	297.36 ± 16.8^b^	104.90 ± 9.37^b,a^
CS300 + TAA	2561.57 ± 57.6^b,a^	319.8 ± 82^b^	129.63 ± 6.16^b^
SY + TAA	2620.77 ± 76.8^b^	348.0 ± 35.3^b^	130.24 ± 5.12^b^

The data were stated as mean ± S.E.M. Means with different superscripts are significantly different. ^a^ *P* < 0.05 versus normal control group and ^b^ *P* < 0.05 versus TAA control group. SY stands for Silymarin (standard hepatoprotective drug).

**Table 4:** Effects of CS extract treatment on the level of MMP-2, MMP-9, and TIMP-1 in the liver tissue at the end of 12 weeks.

Group	MMP-2 (ng/mL)	MMP-9 (ng/mL)	TIMP-1 (ng/mL)
Normal	2.57 ± 0.4^b^	8.31 ± 1.2^b^	1.91 ± 0.79^b^
TAA	8.44 ± 1.06^a^	46.57 ± 4.7^a^	7.81 ± 0.85^a^
CS100	2.44 ± 0.43^b^	8.57 ± 8.11^b^	1.83 ± 0.38^b^
CS300	2.37 ± 0.65^b^	8.8 ± 0.75^b^	2.04 ± 0.67^b^
CS100 + TAA	6.43 ± 0.569^a,b^	22.76 ± 1.78^a,b^	4.78 ± 1.01
CS300 + TAA	4.87 ± 0.77^a,b^	15.51 ± 2.44^a,b^	3.05 ± 0.63
SY + TAA	3.38 ± 0.525^b^	13.84 ± 2.8^a,b^	2.12 ± 0.48^b^

The data were stated as mean ± S.E.M. Means with different superscripts are significantly different. ^a^ *P* < 0.05 versus normal control group and ^b^ *P* < 0.05 versus TAA control group. SY stands for Silymarin (standard hepatoprotective drug).

## References

[1] Ueki T, Kaneda Y, Tsutsui H (1999). Hepatocyte growth factor gene therapy of liver cirrhosis in rats. *Nature Medicine*.

[2] Munoz Torres E, Paz Bouza JI, Lopez Bravo A, Abad Hernandez MM, Carrascal Marino E (1991). Experimental thioacetamide-induced cirrhosis of the liver. *Histology and Histopathology*.

RETRACTED

[3] Schuppan D, Afdhal NH (2008). Liver cirrhosis. *The Lancet*.

[4] Cassiman D, Denef C, Desmet VJ, Roskams T (2001). Human and rat hepatic stellate cells express neurotrophins and neurotrophin receptors. *Hepatology*.

[5] Reid R, Muir R, Levison DA, Burt AD (2008). *Muir's Textbook of Pathology*.

[6] Kadir FA, Kassim NM, Abdulla MA, Yehye WA (2013). Hepatoprotective role of ethanolic extract of vitex negundo in thioacetamide-induced liver fibrosis in male rats. *Evidence-Based Complementary and Alternative Medicine*.

[7] Badami S, Moorkoth S, Suresh B (2004). *Caesalpinia sappan*—a medicinal and dye yielding plant. *Natural Product Radiance*.

[8] Lee JY, Min KJ (2011). Antimicrobial activity and bactericidal activity of *Caesalpinia sappan* L. extract. *Hangug Hwangyeong Bogeon Haghoeji*.

[9] Yodsaoue O, Cheenpracha S, Karalai C, Ponglimanont C, Tewtrakul S (2009). Anti-allergic activity of principles from the roots and heartwood of *Caesalpinia sappan* on antigen-induced *β*-hexosaminidase release. *Phytotherapy Research*.

[10] Moon H-I, Chung I-M, Seo S-H, Kang E-Y (2010). Protective effects of 3'-deoxy-4-omethylepisappanol from *Caesalpinia sappan* against glutamate-induced neurotoxicity in primary cultured rat cortical cells. *Phytotherapy Research*.

[11] Moon CK Drugs from Caesalpinia.

[12] Xu J, Shi T, Zhang S, Guo S, Qiao L, Li K Manufacture and application of water extract of caesalpinia sappan for treating ascites tumor and leukemia.

[13] Park WH, Lee MJ, Kim JY, Jung YH Pharmaceutical composition containing *Caesalpinia sappan* extract for preventing and treating arteriosclerosis.

[14] Hu J, Yan X, Wang W, Wu H, Hua L, Du L (2008). Antioxidant activity *in vitro* of three constituents from *Caesalpinia sappan* L. *Tsinghua Science and Technology*.

[15] Srillakshmi VS, Vijayan P, Raj PV, Dhanaraj SA, Chandrashekhar HR (2010). Hepatoprotective properties of *Caesalpinia sappan* Linn. heartwood on carbon tetrachloride induced toxicity. *Indian Journal of Experimental Biology*.

[16] Sarumathy K, Vijay T, Palani S, Sakthivel K, Rajan MSD (2011). Antioxidant and hepatoprotective effects of *Caesalpinia sappan* against acetaminophen-induced hepatotoxicity in rats. *International Journal of Pharmacology and Therapeutics*.

[17] R Pramely LSR (2012). Prediction of biological activity spectra of a few phytoconstituents of Azadirachta indicia A. Juss. *Journal of Biochemical Technology*.

[18] Lagunin A, Stepanchikova A, Filimonov D, Poroikov V (2000). PASS: prediction of activity spectra for biologically active substances. *Bioinformatics*.

RETRACTED

[19] Ueki T, Kaneda Y, Tsutsui H (1999). Hepatocyte growth factor gene therapy of liver cirrhosis in rats. *Nature Medicine*.

[20] Koehn FE, Carter GT (2005). The evolving role of natural products in drug discovery. *Nature Reviews Drug Discovery*.

[21] (1996). *Guide for the Care and Use of Laboratory Animals*.

[22] Zhao X-Y, Wang B-E, Li X-M, Wang T-L (2008). Newly proposed fibrosis staging criterion for assessing carbon tetrachloride- and albumin complex-induced liver fibrosis in rodents. *Pathology International*.

[23] Kuzu N, Metin K, Dagli AF (2007). Protective role of genistein in acute liver damage induced by carbon tetrachloride. *Mediators of Inflammation*.

[24] Amali AA, Rekha RD, Lin CJ-F (2006). Thioacetamide induced liver damage in zebrafish embryo as a disease model for steatohepatitis. *Journal of Biomedical Science*.

[25] Okazaki I, Ninomiya Y, Kyuichi T, Friedman SI (2003). *Extracellular Matrix and the Liver: Approach to Gene Therapy*.

[26] Kadir FA, Othman F, Abdulla MA, Hussan F, Hassandarvish P (2011). Effect of Tinospora crispa on thioacetamide-induced liver cirrhosis in rats. *Indian Journal of Pharmacology*.

[27] Spira B, Raw I (2000). The effect of thioacetamide on the activity and expression of cytosolic rat liver glutathione-S-transferase. *Molecular and Cellular Biochemistry*.

[28] Bruck R, Aeed H, Shirin H (1999). The hydroxyl radical scavengers dimethylsulfoxide and dimethylthiourea protect rats against thioacetamide-induced fulminant hepatic failure. *Journal of Hepatology*.

[29] Derek GDW (1994). *Systemic Pathology: Liver, Biliary Tract and Exocrine Pancreas*.

[30] Kropacova K, Misurova E, H EH (1998). Protective and therapeutic effect of silymarin on the development of latent liver damage. *Radiatsionnaia Biologiia, Radioecologiia*.

[31] Luper S (1998). A review of plants used in the treatment of Liver disease: part 1. *Alternative Medicine Review*.

[32] Janbaz KH, Gilani AH (2000). Studies on preventive and curative effects of berberine on chemical-induced hepatotoxicity in rodents. *Fitoterapia*.

[33] Nanji AA, Jokelainen K, Tipoe GL, Rahemtulla A, Thomas P, Dannenberg AJ (2003). Curcumin prevents alcohol-induced liver disease in rats by inhibiting the expression of NF-*κ*B-dependent genes. *American Journal of Physiology*.

[34] Agarwal M, Srivastava VK, Saxena KK, Kumar A (2006). Hepatoprotective activity of Beta vulgaris against CCl4-induced hepatic injury in rats. *Fitoterapia*.

[35] Lagunin AA, Gomazkov OA, Filimonov DA (2003). Computer-aided selection of potential antihypertensive compounds with dual mechanism of action. *Journal of Medicinal Chemistry*.

[36] P AV (1998). Computer-assisted mechanism-of action analysis of large databases, including 250,000 open NCI database compounds. *Plant Resources*.

RETRACTED

[37] Moon CK Drugs from Caesalpinia.

[38] Park WH, Lee MJ, Kim JY, Jung YH Pharmaceutical composition containing *Caesalpinia sappan* extract for preventing and treating arteriosclerosis.

[39] Reeves HL, Friedman SL (2002). Activation of hepatic stellate cells—a key issue in liver fibrosis. *Frontiers in Bioscience*.

[40] Yu E, Choe G, Gong G, Lee I (1993). Expression of alpha-smooth muscle actin in liver diseases. *Journal of Korean medical science*.

[41] Sanderson N, Factor V, Nagy P (1995). Hepatic expression of mature transforming growth factor *β*1 in transgenic mice results in multiple tissue lesions. *Proceedings of the National Academy of Sciences of the United States of America*.

[42] Poli G (2000). Pathogenesis of liver fibrosis: role of oxidative stress. *Molecular Aspects of Medicine*.

[43] Zhang B-J, Xu D, Guo Y, Ping J, Chen L-B, Wang H (2008). Protection by and anti-oxidant mechanism of berberine against rat liver fibrosis induced by multiple hepatotoxic factors. *Clinical and Experimental Pharmacology and Physiology*.

[44] Klaunig JE, Kamendulis LM, Hocevar BA (2010). Oxidative stress and oxidative damage in carcinogenesis. *Toxicologic Pathology*.

[45] Park SY, Shin HW, Lee KB, Lee M-J, Jang J-J (2010). Differential expression of matrix metalloproteinases and tissue inhibitors of metalloproteinases in thioacetamide-induced chronic liver injury. *Journal of Korean Medical Science*.

[46] Malhi H, Gores GJ, Lemasters JJ (2006). Apoptosis and necrosis in the liver: a tale of two deaths?. *Hepatology*.

[47] Salama SM, Abdulla MA, AlRashdi AS, Ismail S, Alkiyumi SS, Golbabapour S (2013). Hepatoprotective effect of ethanolic extract of *Curcuma longa* on thioacetamide induced liver cirrhosis in rats. *BMC Complementary and Alternative Medicine*.

[48] Abraham D, Ponticos M, Nagase H (2005). Connective tissue remodelling: cross-talk between endothelins and matrix metalloproteinases. *Current Vascular Pharmacology*.

[49] Wang Y, Zhang J-S, Huang G-C, Cheng Q, Zhao Z-H (2005). Effects of adrenomedullin gene overexpression on biological behavior of hepatic stellate cells. *World Journal of Gastroenterology*.

[50] Parsons CJ, Bradford BU, Pan CQ (2004). Antifibrotic effects of a tissue inhibitor of metalloproteinase-1 antibody on established liver fibrosis in rats. *Hepatology*.

[51] Shi G-F, Li Q (2005). Effects of oxymatrine on experimental hepatic fibrosis and its mechanism in vivo. *World Journal of Gastroenterology*.

[52] An JH, Seong J, Oh H, Kim W, Han KH, Paik YH (2006). Protein expression profiles in a rat cirrhotic model induced by thioacetamide. *The Korean journal of hepatology*.

RETRACTED

[53] Bruck R, Ashkenazi M, Weiss S (2007). Prevention of liver cirrhosis in rats by curcumin. *Liver International*.

